The article "Athlete Behavior Recognition Technology Based on Siamese-RPN Tracker Model" was retracted in 2023. Reasons: unreliable results or conclusions; concerns about the data; concerns about the peer review; concerns about the citations.

# Athlete Behavior Recognition Technology Based on Siamese-RPN Tracker Model

**DOI:** 10.1155/2021/6255390

**Published:** 2021-10-19

**Authors:** Changhui Gao

**Affiliations:** Public Physical Education Department, Xinyang University, Xinyang, Henan 464000, China

## Abstract

With the rapid development of deep learning algorithms, it is gradually applied in UAV (Unmanned Aerial Vehicle) driving, visual recognition, target tracking, behavior recognition, and other fields. In the field of sports, many scientists put forward the research of target tracking and recognition technology based on deep learning algorithms for athletes' trajectory and behavior capture. Based on the target tracking algorithm, a regional proposal network RPN algorithm combined with the twin regional proposal network Siamese algorithm is proposed to study the tracking and recognition technology of athletes' behavior. Then, the adaptive updating network is used to track the behavior target of athletes, and the simulation model of behavior recognition is established. This algorithm is different from the traditional twin network algorithm. It can accurately take the athlete's behavior as the target candidate box in model training and reduce the interference of environment and other factors on model recognition. The results show that the Siamese-RPN algorithm can reduce the interference from the background and environment when tracking the athletes' target behavior trajectory. This algorithm can improve the training behavior recognition model, ignore the background interference elements of the behavior image, and improve the accuracy and overall performance of the model. Compared with the traditional twin network method for sports behavior recognition, the Siamese-RPN algorithm studied in this paper can perform offline operations and distinguish the interference factors of athletes' background environment. It can quickly capture the characteristic points of athletes' behavior as the data input of the tracking model, so it has excellent popularization and application value.

## 1. Introduction

In recent years, the target behavior tracking model and behavior recognition technology are the important direction of the development of the artificial intelligence deep learning network [1]. With the distinction between supervised and unsupervised deep learning algorithms, deep learning algorithms are widely used in security protection, driverless, smart home, public transportation, sports, and other fields [2, 3]. In the field of sports, the demand for athletes' behavior trajectory analysis and behavior pattern recognition is gradually increasing [4]. In the traditional single-target tracking model, many researchers use the athletes' position of the initial video frames per time for behavior trajectory analysis [5] and according to the athlete's characteristic points to identify the action behavior. However, the traditional single target tracking algorithm cannot accurately capture the moving position, and the tracking target model often shows deformation, speed of control, many interference factors, and other reasons [6]. This situation makes the tracking model cannot accurately capture the trajectory and the position of feature points in the process of athletes' behavior tracking and recognition [7, 8]. It cannot complete the purpose of accurate behavior recognition. Follow-up researchers proposed a mean-based tracking algorithm, which does not need data validation, and only needs tracking modeling of the athlete's target to achieve iterative search to determine the target position [9]. This algorithm has fast iteration speed and high computational efficiency, but its persistence is poor, and its accuracy cannot be guaranteed [10]. The results of behavior recognition cannot be accurately captured when the target motion is deformed. One after another, the method of using correlation over filtering to calculate target tracking and recognition has gradually become the mainstream mode [11]. In this way, the information data is combined with the tracking model for the first time, and the correlation filter is used to detect the responsiveness in the frame number of the behavior of the moving person, and the feature points of the data are captured. It further improves the recognition efficiency of the tracking model, and the speed can exceed 100 frames [12, 13].

The article "Athlete Behavior Recognition Technology Based on Siamese-RPN Tracker Model" was retracted in 2023. Reasons: unreliable results or conclusions; concerns about the data; concerns about the peer review; concerns about the citations.

In recent years, with the rapid development of deep learning algorithms in the field of computers, vision, and recognition [14], many researchers apply the convolutional neural network algorithm to classification function, which can extract a large number of feature points to train the tracking model, so as to improve the performance of behavior recognition model [15]. In the deep learning algorithm, the twin network has the characteristics of sharing data, which is suitable for repetitive similar processing tasks. Siamese FC, a twin network target tracking algorithm, can combine the number of video frames with the feature points extracted by the convolution network to obtain the predicted position of target behavior [16]. Subsequently, based on the above tracking model behavior recognition technology development, this paper proposes the Siamese-RPN algorithm, which can accurately identify the candidate box of athletes' behavior target and reduce the influence of environmental factors on Athletes' behavior recognition model [17–19].

The article "Athlete Behavior Recognition Technology Based on Siamese-RPN Tracker Model" was retracted in 2023. Reasons: unreliable results or conclusions; concerns about the data; concerns about the peer review; concerns about the citations.

Contributions in this paper are summarized as follows: (1) a regional proposal network RPN algorithm combined with the twin regional proposal network Siamese algorithm is proposed to study the tracking and recognition technology of athletes' behavior; (2) the proposed model can accurately take the athlete's behavior as the target candidate box in model training and reduce the interference of environment and other factors on model recognition; and (3) compared with the traditional twin network method for sports behavior recognition, the proposed model in this paper can perform an offline operation and distinguish the interference factors of athletes' background environment. It can quickly capture the characteristic points of athletes' behavior as the data input of the tracking model, so it has excellent popularization and application value.

The following content is divided into four sections. The first section introduces the related work about the development of tracking model technology and behavior recognition technology. The second section discusses the Siamese-RPN algorithm to study the target tracking model and athlete behavior recognition technology. Firstly, the proposed tracking algorithm by probability regression and the proposed athlete behavior tracking recognition model are optimized. Finally, an adaptive updating algorithm is proposed to build a tracker model, and the simulation model of athlete behavior recognition is established. The third section is the result analysis on the Siamese-RPN algorithm for athlete target tracking. The fourth section is the conclusion to output some important results.

## 2. Related Work

Athlete behavior recognition is a part of the application of the tracker model in the field of artificial intelligence recognition [20]. Firstly, the target tracking algorithm in the tracker model is used to capture the behavior trajectory of the moving person, and finally, the simulation model is constructed by using behavior recognition technology [21]. In athlete target tracking, it is necessary to predict the change of target position in each frame number, but in the tracking process, there will be occlusion, size change, deformation, complex background, illumination, and other influencing factors [22]. To realize the recognition of behavior, we must first solve the problem of target tracking and capture. In recent years, target tracking is based on the Siamese twin network framework. The core content is to capture the repetitive similar actions in the search area according to the learning training template and matching rules [23]. However, the common network algorithm will consume tracking time and the tracking target is not accurate. Based on the common network, many subsequent researchers proposed the introduction of the region proposal algorithm to obtain a more accurate target range [24]. The tracker model constructed by the Siamese-RPN algorithm can accurately capture the target behavior box and reduce the influence factors of complex background. Through the classification and regression branch of target tracking, finally build the behavior recognition model of athletes.

The article "Athlete Behavior Recognition Technology Based on Siamese-RPN Tracker Model" was retracted in 2023. Reasons: unreliable results or conclusions; concerns about the data; concerns about the peer review; concerns about the citations.

Xu et al. invested a lot of research energy and funds in tracking technology and behavior recognition technology [25]. With the large demand for target tracking technology, the deep learning algorithm is also improving. They focused on the research and development of target tracking and monitoring projects, mainly applied in the battlefield and civil environment. After the real-time monitoring model is established, human behavior tracking and capturing is realized. And it can identify whether people carry dangerous goods and other functions.

Deng et al. mainly applied target tracking and behavior recognition technology in the public transport monitoring system, aiming at tracking and interactive recognition of people's traffic behavior and vehicle driving [26]. They combined the deep learning algorithm with the feature point analysis technology to form the ability to accurately track illegal vehicle behavior in a complex environment, as well as the realization of the illegal personnel behavior identification. After analysis and identification, the violation information is uploaded to the management and control system.

Jia et al. also applied tracking technology to traffic management. They mainly implanted the tracking algorithm and recognition algorithm into the radar system [27]. Through the target tracking and behavior recognition control of traffic vehicles, it can achieve the measurement of vehicle distance, angle, speed, and other functions. Later, they also used this technology in the VR model. In the virtual environment, eye movement is tracked and real-time interaction is realized.

Visual tracking and behavior recognition are applied in automation, medical image, artificial intelligence, and other fields [28]. This paper mainly studies the classification and behavior understanding of the target in the tracking model. The function of human body recognition and motion tracking is realized. The development of this technology is conducive to the optimization of the public security environment of the whole society. According to the application and development of target tracking and behavior recognition technology in the above countries, this paper studies the tracking technology and finally realizes the establishment of the athlete's behavior recognition model. In the tracking model, the target personnel is locked and tracked, and then the Siamese-RPN algorithm is optimized to improve the tracking speed and performance. Finally, the Siamese-RPN algorithm adaptive update tracking technology combined with the behavior recognition of sports personnel is used to build the simulation model.

The article "Athlete Behavior Recognition Technology Based on Siamese-RPN Tracker Model" was retracted in 2023. Reasons: unreliable results or conclusions; concerns about the data; concerns about the peer review; concerns about the citations.

## 3. Methods on Athlete Behavior Recognition Technology based on Siamese-RPN Network Tracking Model

### 3.1. Method on Athletes' Behavior Locking and Target Tracking Technology based on Siamese-RPN Network

Twin network is composed of two or more network structures in the deep learning network algorithm, which can be calculated according to a variety of input variables. And it can share the weight in the network structure. The core content of the twin network is to find a group of variables and find the variables of similarity by specifying the spatial range between target distances [29]. It makes the difference between the degree values of variables in the same class smaller and the difference between different classes larger. The traditional target tracking behavior recognition technology uses the Siamese FC algorithm, a twin network structure tracking model based on all connected layers. The core of the algorithm is to compare the similarity between the original sample image and the target image through the training function. If the similarity of target judgment is consistent, the score is higher; otherwise, it is lower. However, this algorithm cannot guarantee high performance in accuracy, and it will show the problem of tracking target deformation and will be interfered with by various backgrounds and environments. Based on the above situation, this paper proposes the Siamese-RPN algorithm to integrate the candidate networks into an architecture and uses the RPN attention mechanism and frame regression classification to screen out background and environmental interference factors. The structure of the twin network area proposal algorithm is shown in Figure 1.

As can be seen from Figure 1, the Siamese-RPN network can realize offline training operation between end-to-end models. This structure is divided into many branches, the original target and the tracking target are classified into two paths, and the twin network is used to extract network feature points to achieve the function of target recognition. The multirange evaluation mechanism and online strategy of traditional tracking technology are changed, and the tracking technology is improved to a detection process for a certain target. The performance and detection efficiency of the whole tracking model are improved. In the offline operation, the target position is predicted and located by the loss function and the repeated range of the set threshold value, and the target area is screened. The loss function formula is as follows:

(1) $$\begin{array}{c} l_{\text{total}}=\alpha \sum_{i=1}^{3}l_{\text{cls}}+\beta \sum_{i=1}^{3}l_{\text{reg}},\\ l_{\text{cls}}=\frac{-\sum_{i}^{n}{\text{labels}}_{i}\cdot \mathrm{lg}\left({\text{scores}}_{i}\right)}{n},\\ l_{\text{reg}}=\frac{-\sum_{i}^{n}\sum_{j}^{4}R\left(t_{j}-t_{j}^{*}\right)}{n}. \end{array}$$

The weight coefficient of loss is defined in the formula, and the background environmental factors are classified into two categories. The loss coefficient of the bounding box is updated, and the number of effective mechanism variables in the candidate region is selected for calculation. The threshold of intersection and union differentiation is set as the range of matching parameters. Different thresholds will affect the prediction range and border regression of the tracking target:

(2) $$\begin{array}{c} \text{IOU}=\frac{\text{area}\left(C\right)\cap \text{area}\left(G\right)}{\text{area}\left(C\right)\cup \text{area}\left(G\right)}. \end{array}$$

The process of athlete behavior recognition is a process of target location and tracking. Firstly, each video material is divided into any number of frames. And the motion state of each frame position is predicted. The simplest operation is to track the range of the target according to the shape box. The flow of the target tracking algorithm is shown in Figure 2.

The article "Athlete Behavior Recognition Technology Based on Siamese-RPN Tracker Model" was retracted in 2023. Reasons: unreliable results or conclusions; concerns about the data; concerns about the peer review; concerns about the citations.

When tracking and identifying athletes' behavior, if the target has other positioning, the tracking task can be defined as a regression calculation process. We need to build a model to track the position and analyse the state of the target. The traditional tracking model uses confidence regression to optimize the operation, that is to predict the similarity between the feedback state feature and the target feature. This method is mainly used in the deep learning algorithm and mainstream tracking method, and our regression algorithm can predict the trajectory of an independent target [30]. In the regression algorithm, the background interference in the traditional tracking can be ignored, and the appropriate prediction method can be improved. In the process of athlete's behavior locking, if the target changes, the position of the center shape box will be different from that of the target center, as shown in Figure 3.

It can be seen from Figure 3 that the general regression algorithm can only focus on a single target, ignoring the gap between the shape box positions, which is not conducive to the target tracking task. Therefore, this paper proposes to solve the location difference problem in Siamese-RPN by using the shape box of the probability regression algorithm. The node with the largest probability density is selected as the prediction output, that is, the target center position. When training the Siamese-RPN network, the prediction probability distribution of input data and output data is calculated firstly:

(3) $$\begin{array}{c} p\left(y|x,\theta \right)=\frac{1}{z_{\theta }\left(x\right)}e^{s\theta \left(y,x\right)},\\ z_{\theta }\left(x\right)=\int e^{s\theta \left(y,x\right)}\text{d}y. \end{array}$$

Because the *sθ*(*y*, *x*) parameter is essentially converted from the confidence number, that is to say, the relationship between input data and output data is a standard value, the purpose of the above formula is to convert the value into probability density. Finally, it is adjusted by function normalization. In view of the difference between the conditional distribution described by the negative likelihood number and the conditional probability distribution predicted by the negative likelihood number, we use the divergence transformation to define it [31]:

(4) $$\begin{array}{c} D_{KL}\left(p\|q\right)=\sum_{i=1}^{N}p\left(x_{i}\right)\log\left(\frac{p\left(x_{i}\right)}{q\left(x_{i}\right)}\right). \end{array}$$

In the formula, *q*(*x*_*i*_) is the target approximate distribution and *p*(*x*_*i*_) is the real location distribution [32]. After the divergence variable is defined, the training network parameters can be calculated:

(5) $$\begin{array}{c} KL\left(p\left(\cdot |y_{i}\right),p\left(\cdot |x_{i},\theta \right)\right)=\int p\left(y|y_{i}\right)\log\frac{p\left(y|y_{i}\right)}{p\left(y|x_{i,\theta }\right)}\text{d}y,\\ KL\left(p\left(\cdot |y_{i}\right),p\left(\cdot |x_{i},\theta \right)\right)=\log\left(\int e^{s\theta \left(y,x_{i}\right)}\text{d}y\right)-\int s_{\theta }\left(y,x_{i}\right)p\left(y|y_{i}\right)\text{d}y. \end{array}$$

By minimizing the value of output divergence, the most accurate value of probability prediction distribution can be obtained. The comparison between the actual accuracy and the prediction accuracy of the probability regression algorithm in the Siamese-RPN network is shown in Figure 4.

The article "Athlete Behavior Recognition Technology Based on Siamese-RPN Tracker Model" was retracted in 2023. Reasons: unreliable results or conclusions; concerns about the data; concerns about the peer review; concerns about the citations.

As can be seen from Figure 4, with the increase of the number of training iterations, the accuracy also gradually increases. The final result accuracy of the Siamese-RPN algorithm is basically close to the prediction result. In conclusion, the tracker model based on the Siamese-RPN network can improve the accuracy of athletes' behavior tracking and recognition.

### 3.2. Method on Athlete Behavior Tracking and Recognition Technology based on Adaptive Update of Siamese-RPN Network

Compared with the traditional twin network algorithm, the Siamese-RPN network can take into account the influence factors of the background environment information in the process of behavior tracking and recognition and has a stronger discrimination ability in the face of interference information. Therefore, this paper proposes an adaptive target classification updating behavior tracking algorithm based on the Siamese-RPN network. To accurately obtain the target motion position, the cross-correlation feature monitoring module is introduced. The offline training and learning method is used to supervise the behavior recognition feature points of athletes. Finally, the attention mechanism is introduced to analyse the background environment information in the video image, to extract the accurate target feature point information. The update mechanism is mainly divided into two modules: the judgmental target classification module and the adaptive module. Through feature point information extraction, Siamese-RPN algorithm model, classification and supervision feature point model, adaptive model, and so on, the athlete behavior recognition model is constructed.

Based on the Siamese-RPN algorithm, the best matching box position in the region to be searched is calculated by training and learning embedded spatial feature point extraction model. The calculation formula is as follows:

(6) $$\begin{array}{c} f_{M}\left(x,z\right)=\varphi \left(x\right)*\varphi \left(Z\right)+b*1. \end{array}$$

In the formula, the branch variable is used to learn the feature point representation of the training target module, and the other branch variable is used in detection. The network parameter weights of the two branches are shared. Based on this formula, the defined variables in the candidate network are used to calculate the predicted target position and boundary box independently. The formula is as follows:

(7) $$\begin{array}{c} f_{M}^{\text{cls}}\left(x,z\right)=h^{\text{cls}}\left[\varphi_{\text{cls}}\left(x\right)*\varphi_{\text{cls}}\left(z\right)\right],\\ f_{M}^{\text{reg}}\left(x,z\right)=h^{\text{reg}}\left[\varphi_{\text{reg}}\left(x\right)*\varphi_{\text{reg}}\left(z\right)\right]. \end{array}$$

The independent variables are used to learn the feature point representation of the original template frame and the detection frame and store the background information of each definition box. *f*_*M*_^reg^(*x*, *z*) stores the width height ratio information between the offset coordinates of the center box point of the prediction definition and the real box. It can get more accurate background score information of the moving target. On this basis, the boundary box regression calculation is carried out for the center point with the highest score:

(8) $$\begin{array}{c} B_{\text{predict}}=\left(x^{\text{pre}},y^{\text{pre}},w^{\text{pre}},h^{\text{pre}}\right),\\ x^{\text{pre}}=\overset{\wedge \text{an}}{x}+\text{d}x^{\text{reg}}\cdot \overset{\wedge \text{an}}{w},\\ y^{\text{pre}}=\overset{\wedge \text{an}}{y}+\text{d}y^{\text{reg}}\cdot \overset{\wedge \text{an}}{h},\\ w^{\text{pre}}=\overset{\wedge \text{an}}{w}+e^{\text{d}w^{\text{reg}}},\\ h^{\text{pre}}=\overset{\wedge \text{an}}{h}+h^{\text{d}h^{\text{reg}}}. \end{array}$$

After the final boundary frame coordinates of target position prediction are calculated according to the above formula, we need to compare the local similarity between the template frame and detection frame based on the Siamese-RPN network target tracking algorithm. The top position of the cross-correlation feature map is the actual coordinate of the target to be tracked. The RPN module can get an efficient and accurate image when it is modified.

The article "Athlete Behavior Recognition Technology Based on Siamese-RPN Tracker Model" was retracted in 2023. Reasons: unreliable results or conclusions; concerns about the data; concerns about the peer review; concerns about the citations.

The image change is related to the corresponding weight value in the RPN module. In the training, we also need to train and learn the weight value. In the athlete behavior recognition model, it is necessary to set the target classification module and extract the target feature points for training. The attention mechanism is used to analyse the two-dimensional spatial feature map, and the weight coefficient of coordinate position is obtained. Finally, the feature information of the corresponding target is extracted to separate the tracking target from other interference factors in the region. The comparative analysis of the number of feature points extracted by the Siamese-RPN algorithm and traditional tracking algorithm on the accuracy coefficient of the target position is shown in Figure 5.

It can be seen from Figure 6 that the tracking model using Siamese-RPN is more accurate than the traditional tracking algorithm in target behavior recognition and tracking with the increase of the number of feature points extracted. In the above adaptive update strategy, the original information of the target is accumulated according to the initial frame number, and the predicted current position is compared with the extracted template information. The results show that the adaptive updating model can capture and transmit the deep feature points in the current region. The real motion behavior of the first time is fed back to the target bounding box, which is based on the twin region proposed algorithm to predict the final target behavior model. The results show that the adaptive updating strategy based on Siamese-RPN can recognize and track the behavior of athletes under the interference of many factors.

The article "Athlete Behavior Recognition Technology Based on Siamese-RPN Tracker Model" was retracted in 2023. Reasons: unreliable results or conclusions; concerns about the data; concerns about the peer review; concerns about the citations.

In the process of athlete behavior recognition, it is necessary to analyse the contour of the human body. It will change regularly according to the time factor. The description of athletes' behavior has obvious representativeness, and the analysis of behavior contour can be carried out according to the shape, movement rules, and other aspects. After extracting the behavior contour from the video image data, the boundary extraction method is used to capture the coordinate points. After getting the center coordinates of the detailed position, the maximum pixel is taken as the starting point, and the whole scope box is obtained by rotating in the direction. To eliminate the influence factors in the process of recognition, it is necessary to standardize the image. The number of data points affects the distance distribution of the overall feature points. The comparison of the results before and after the standardized processing is shown in Figure 6.

It can be seen from Figure 6 that the distance distribution curve of the feature points after the standardization treatment is obviously more simplified than that before the treatment. It can eliminate the interference feature factors in the whole recognition process.

## 4. Results Analysis on Athlete Behavior Recognition Technology Based on Siamese-RPN Network Tracking Model

### 4.1. Results of Athletes' Behavior Locking and Target Tracking Based on Siamese-RPN Network

The whole algorithm uses the data source set of athletes' sports as training data, video information, and image information of totally more than 5000 groups of data. The sample data is trained and tested respectively, and the edge of each frame in the video data is cut and filled. The pixel definition of image information is guaranteed. Firstly, the Siamese-RPN algorithm is used to train the model offline, and then target tracking is carried out. In the training environment, the data is preprocessed and the network structure is simplified. It is necessary to model from the center coordinates of the first frame and the target box when capturing the athlete's behavior target. Finally, the output data is trained by a regression model to get the behavior goal of athletes after removing the interference factors. In the whole experiment, we detect and analyse the center position error and overlap rate and calculate the accuracy difference between the Siamese-RPN algorithm and the traditional tracking algorithm. The change of accuracy under the influence of the center position threshold is shown in Figure 7. The change of accuracy under the influence of overlap rate is shown in Figure 8.

The article "Athlete Behavior Recognition Technology Based on Siamese-RPN Tracker Model" was retracted in 2023. Reasons: unreliable results or conclusions; concerns about the data; concerns about the peer review; concerns about the citations.

It can be seen from Figure 8 that the number of target frame center position errors calculated by the Siamese-RPN algorithm has little effect on the accuracy. With the increase of the error threshold, the accuracy of the traditional algorithm decreases obviously. As can be seen from Figure 9, the influence of overlap rate on both algorithms is obvious. Compared with the expected curve, the accuracy based on the Siamese-RPN algorithm can keep in the same range of the prediction curve under the influence of the overlap rate. In conclusion, the athlete behavior locking and target tracking technology based on the Siamese-RPN algorithm has good performance.

### 4.2. Results of Athletes' Behavior Tracking and Recognition Based on Adaptive Update of Siamese-RPN Network

To verify the effectiveness of the tracking method based on the adaptive update of the Siamese-RPN network, the artificially labelled image data set is supplemented with tracking points, mainly from the camera movement, athletes' behavior track, light changes, shelter, and other aspects of supplement. For different motion recognition, using different parameters to calculate can get the maximum performance comparison results. Therefore, this paper uses the control variable method to evaluate the parameter data and find the most suitable parameter range for the experiment. The optimized data set can reduce the waste of time of the identification model. The evaluation data is introduced into the cross-correlation feature map to update the monitoring module, classification module, and adaptive module. This paper analyses the data quantity and recognition success rate of the adaptive strategy model using the Siamese-RPN algorithm and finally compares it with the ordinary tracking algorithm without the Siamese-RPN algorithm. The change of contrast curve is shown in Figure 9.

Siamese-RPN can still maintain the success rate of recognition when the amount of input data increases. Compared with the traditional tracking algorithm, the performance has been greatly improved. In the athlete behavior recognition model, the feature points extracted from the contour can ensure that the processed image is clear and accurate, which ensures the recognition efficiency and accuracy of the model. In the analysis of athletes' behavior, whether there is contour analysis can determine the result of behavior recognition. Therefore, this paper proposes to use the Siamese-RPN algorithm to track athletes' behavior and obtain athletes' feature points according to the contour to supplement the recognition model.

The article "Athlete Behavior Recognition Technology Based on Siamese-RPN Tracker Model" was retracted in 2023. Reasons: unreliable results or conclusions; concerns about the data; concerns about the peer review; concerns about the citations.

## 5. Conclusions

With the extensive application of deep learning algorithms in automobile driving, traffic management, artificial intelligence, and pattern recognition, many tracking algorithms have been produced for pattern recognition. In many tracking algorithms, the traditional Siamese FC network algorithm cannot meet the needs of target tracking and recognition. This algorithm will be affected by many factors such as background and environment and cannot guarantee the accuracy of target recognition and detection. Based on the target tracking algorithm, this paper proposes an algorithm based on the RPN tracker model to track and recognize athletes' behavior. This algorithm can optimize the original tracking model and eliminate the influence of interference factors. By changing the training model to offline mode, the original target area can be distinguished, and the bounding box is defined to track the target behavior. Firstly, the probability regression algorithm is used to classify the background factors to optimize the location accuracy of target tracking in the athlete behavior recognition. The results show that the Siamese-RPN algorithm has more accurate ability to capture the target than the traditional tracking algorithm and can clearly identify the behavior of athletes. Finally, this algorithm is combined with the adaptive update strategy to change the capture mode of behavior recognition feature points. The results show that the efficiency of feature point capture based on the Siamese-RPN algorithm increases with the increase in input data. In the process of athlete behavior recognition, the overall recognition success rate is improved.

## Figures and Tables

**Figure 1:** Structure chart of twin network area proposal algorithm.

**Figure 2:** Flowchart of the target tracking algorithm.

**Figure 3:** Comparison between target box and target center.

**Figure 4:** Comparison chart of actual accuracy and prediction accuracy of calculation results in the Siamese-RPN network.

**Figure 5:** Comparison of precision coefficients between the Siamese-RPN algorithm and traditional tracking algorithm.

**Figure 6:** Comparison of results before and after standardization.

**Figure 7:** Accuracy change of two algorithms under the influence of center position threshold.

**Figure 8:** Comparison of the accuracy of the two algorithms under the influence of overlap rate.

**Figure 9:** Comparison of recognition success rate between the Siamese-RPN algorithm and ordinary tracking algorithm.

## Data Availability

The data used to support the findings of this study are available from the corresponding author upon request.
